# Effect of Tongluozhitong Prescription-Assisted Intra-Articular Injection of Sodium Hyaluronate on VAS Score and Knee Lysholm Score in Patients with Knee Osteoarthritis

**DOI:** 10.1155/2021/3210494

**Published:** 2021-10-28

**Authors:** Jianfang Gong, Qiang Li, Mengling Wei, Liangliang Xue, Yinlian Liu, Jun Gao, Tiantian Qin

**Affiliations:** ^1^Department of Traditional Chinese Medicine, Bethune Hospital, Taiyuan, Shanxi 030032, China; ^2^Department of Orthopaedics, Bethune Hospital, Taiyuan, Shanxi 030032, China; ^3^Department of Radiology, Bethune Hospital, Taiyuan, Shanxi 030032, China; ^4^Department of Rehabilitation, Bethune Hospital, Taiyuan, Shanxi 030032, China

## Abstract

Knee osteoarthritis (KOA) has become one of the leading causes of workforce loss in the middle-aged and elderly population and a global public health problem second only to cardiovascular disease, so we need to find more effective treatments for this disease. In this study, we selected 120 patients with KOA admitted to our hospital from June 2018 to December 2020 and divided them into treatment group 1, treatment group 2, and joint group according to the random number table method, with 40 patients in each group. Treatment group 1 was treated with Tongluozhitong prescription dip-soaking therapy, treatment 2 group was treated with intra-articular injection of sodium hyaluronate, and the joint group was treated with a combination of both modalities for 4 weeks in all three groups. Clinical efficacy, visual analogue scale (VAS), Lysholm knee score (LKS), activity of daily living score (ADL), the levels of bone metabolic markers such as cartilage oligomeric matrix protein (COMP), type II collagen degradation maker (CTX-II), and matrix metalloproteinase-3 (MMP-3), and the levels of inflammatory mediators such as interleukin-1*β* (IL-1*β*), tumor necrosis factor-*α* (TNF-*α*), and hypersensitive C-reactive protein (hs-CRP) were used as observations to compare and analyze the therapeutic effects of the three treatment regimens in KOA patients. The results showed that the clinical excellence rates of the joint group, treatment group 1, and treatment group 2 were 72.50%, 50.00%, and 90.00%, respectively, with statistically significant differences between any two comparisons. After treatment, VAS scores, serum COMP, CTX-II, MMP-3, IL-1*β*, TNF-*α*, and hs-CRP levels decreased in all three groups, and the levels of each index were as follows: joint group < treatment group 1 < treatment group 2, and the difference between any two comparisons was statistically significant. The LKS score and ADL score increased in all three groups, and the levels of each index were as follows: joint group > treatment group 1 > treatment group 2, with statistically significant differences in any two groups compared. None of the patients in the three groups experienced any significant adverse effects during treatment. This suggests that the dip-soaking therapy of Tongluozhitong prescription is more advantageous than intra-articular sodium hyaluronate injection treatment in suppressing the level of serum bone metabolic markers and inflammatory mediators, reducing pathological joint damage, relieving symptoms of pain, alleviating degenerative joint symptoms, and improving knee function in KOA patients. The combination of the two in KOA patients can significantly improve the efficacy and has a good safety profile.

## 1. Introduction

Knee osteoarthritis (KOA) is a chronic joint disease characterized by deformation and destruction of articular cartilage and osteophytes, which can cause joint pain and dysfunction and seriously affect the quality of life of patients, and is one of the chronic diseases commonly seen in middle-aged and elderly people [1]. The incidence of KOA is increasing year by year with the aging trend of our population, which brings about a great economic burden to the patients themselves, their families, and the society [2]. The pathogenesis of KOA is not well understood and clinical management of the disease focuses on controlling pain, reducing disability, improving knee function, and improving quality of life [3]. There are various treatment modalities for KOA, including oral drugs, topical drugs, intravenous input, and intra-articular injection of drugs, among which intra-articular injection of sodium hyaluronate is currently the most widely used clinical treatment method [4].

Sodium hyaluronate is the main component of synovial fluid and one of the components of cartilage matrix. It can play a lubricating role to reduce the friction between the tissues in the joint cavity after the injection into the joint cavity; it can also promote synovial cells to synthesize polymeric hyaluronic acid to increase the concentration and molecular weight of sodium citrate in the joint fluid and change the viscosity of the joint fluid. In addition to protecting joint cartilage and promoting healing and regeneration of joint cartilage, sodium hyaluronate can also significantly improve the inflammatory response of tissues, relieve pain, and improve joint function [5, 6]. KOA belongs to the category of “rheumatism” in traditional Chinese medicine. Sweating when wind, sitting on wet ground, wading through water and rain, etc., can cause wind, cold and dampness, and other evils to invade the body's meridians and stay in joints, vitrous resulting in obstruction of meridian qi and blood. Therefore, Chinese medicine often uses the principle of warming the meridians, dispersing cold, and relieving pain as treatment [7]. The external treatment method of Chinese medicine emphasizes internal and external application to the organism through different ways, which can achieve the purpose of supporting the righteous energy and eliminating the evil energy, and has extensive clinical experience in the treatment of rheumatism. Chinese medicine dip-soaking therapy is a kind of wet compression method, which is a method to grind the drug and put it in a bag and soak it in the liquid, warm it, and then take it out and apply it wet on the affected area and maintain the temperature by heating it with electromagnetic wave therapeutic apparatus. It has the advantages of exact efficacy, simplicity, and ease of use, as well as few side effects, and is widely used in clinical practice [8].

In this study, we selected the dip-soaking therapy of Tongluozhitong prescription, intra-articular injection of sodium hyaluronate, and the combined application of the two treatments and conducted a comparative analysis of the efficacy of different treatment methods to clarify the effect of combined treatment on the clinical efficacy of KOA patients and provide some reference for the selection of more appropriate treatment methods for KOA patients.

## 2. Materials and Methods

### 2.1. Materials

120 patients with KOA who were admitted to our hospital from June 2018 to December 2020 were selected; among them, 51 males and 69 females were aged from 41 to 70 years, and the mean age was 54.23 ± 7.78 years; the duration of the disease ranged from 5 months to 7 years, with a mean of 3.21 ± 1.36 years. After enrollment, each subject was numbered sequentially (1 to 120). The total number of cases was set at 120 and the number of treatment groups was set at 3 by the random number table method, and the patients were divided into treatment group 1, treatment group 2, and joint group, with 40 cases in each group. The comparison of general data such as gender, age, disease duration, and lesion site in the three groups is shown in Table 1.

### 2.2. Diagnostic Criteria [9]

The diagnostic criteria were as follows: ① recurrent knee pain within the last 1 month which prevents normal work or labor; ② X-ray examination showing that the knee joint space became narrow, osteophytes formed on the edges of the joints, and bone sclerosis or cystic changes appeared under the cartilage; ③ middle-aged and elderly people aged ≥40 years; ④ joint stiffness in the morning ≤30 min; and ⑤ existence of a distinct sensation of bone friction at the affected joint when moving. If ① + ② or ① + ③ + ④ + ⑤ of the diagnostic criteria were met, the diagnosis of KOA was made.

### 2.3. Inclusion Criteria

The inclusion criteria were as follows: ① patients who met the above diagnostic criteria and were diagnosed with KOA; ② patients with joint pain and dysfunction caused by KOA; ③ patients without significant heart, brain, kidney, or lung insufficiency; ④ exclusion of rheumatoid arthritis and other diseases by laboratory tests; ⑤ patients who voluntarily participated in the trial and signed an informed consent form; and ⑥ patients in the age range of 40 to 70 years.

### 2.4. Exclusion Criteria

The exclusion criteria were as follows: ① patients combined with sprains or other traumas; ② those with coexisting severe visceral pathologies or other comorbidities affecting the knee joint, such as psoriasis, syphilitic neuropathy, metabolic bone disease, and gout lesions; ③ patients with serious organic diseases, pregnant women, patients with coagulation disorders, and patients with diabetes mellitus; ④ those with skin problems at the knee joint and poor skin sensation; and ⑤ those who were unable to adhere to the treatment or dropped out in the middle of the treatment for various other reasons and could not judge the efficacy of the treatment.

### 2.5. Treatment Methods

1. Treatment group 1 was treated by dip-soaking with Tongluozhitong prescription, and the specific operations were as follows: 30 g of frankincense, 30 g of myrrh, 30 g of garden balsam stem, 30 g of *Zanthoxylum bungeanum* Maxim., 30 g of radix puerariae, and so forth were put into a cloth bag of about 15 × 20 cm sewn with a towel and soaked in a thermostat for 1 hour and heat to about 40°C and then taken out and wet-applied to the knee joint, and the treatment was administered for 30 minutes under the thermostatic control of the electromagnetic therapy instrument at a temperature of 32 to 45°C (the temperature should be comfortable and tolerable to the patient), 1 time per day for 4 weeks as a course of treatment.
2. Treatment group 2 was treated with intra-articular injection of sodium hyaluronate, and the specific operations were as follows: the patient was treated in a supine position, keeping the knee joint flexed at 45°, and the Neixiyan point (the Neixiyan point is located at the inner depression of the anterior patellar ligament of the knee joint) was selected for routine disinfection and anesthesia. A 5 mL disposable syringe was inserted into the joint cavity to completely extract the fluid from the cavity, without removing the needle, a sodium hyaluronate syringe was attached directly, and 2 mL of sodium hyaluronate was injected slowly and evenly. After the injection was completed, the needle was removed, a band-aid was applied externally, and the patient was allowed to move the knee joint several times to evenly distribute the injection solution, 1 time per week, for a total of 4 treatments.
3. The joint group was treated with a regimen of dip-soaking with Tongluozhitong prescription-assisted intra-articular injection of sodium hyaluronate: the patients in this group were treated for the same duration as the other two groups, for a total of 4 weeks. On the first day of each week, patients were treated by dip-soaking with Tongluozhitong prescription for 30 minutes (same operation as treatment group 1), followed by intra-articular injection of sodium hyaluronate (same operation as treatment group 2), and, starting from the second day of this week, the traditional Chinese medicine dip-soaking therapy treatment was performed only once a day until the end of this week. This cycle was used to complete the subsequent three weeks of treatment.

### 2.6. Observation Indicators

1. Visual analogue scale (VAS) was rated before and after treatment in the three groups, and the scoring criteria were as follows: the VAS score was based on 11 numbers from 0 to 10 representing different levels of pain, where 0 means no pain and 10 means extreme pain, and patients were asked to select a number from the table to represent their pain level before treatment and after 4 weeks of treatment, respectively. A score of 0 indicated that the patient did not feel any pain; 1∼3 indicated mild pain, and the patient's activities were not restricted and did not affect work and life; 4∼6 indicated moderate pain, and the patient's activities were slightly restricted and affected general work and life; 7∼10 indicated severe pain, and the patient's activities were significantly restricted and significantly affected work and life.
2. Patients were rated on knee function before and after treatment using the Lysholm knee scale (LKS): this scale included eight entries for claudication, interlocking, pain, bracing, instability, swelling, stair climbing, and squatting, with a total score of 0 to 100, and the score was proportional to the patient's joint function. The patients' knee function was evaluated before treatment and after 4 weeks of treatment, respectively; a score of >84 indicated normal joint function; a score of 66–84 indicated fair joint function; and a score of ≤65 indicated poor joint function.
3. The activities of daily living (ADL) scale: patients' ADL was assessed before and after treatment using the Barthel Index, one of the most common methods used to assess ADL, which includes 10 items such as eating, bowel control, activity, transfer, bathing, and dressing. The scores for bathing and grooming were 0 and 5; for eating, dressing, bowel control, urine control, toileting, and stairs they were 0, 5, and 10; and for transfer and activities they were 0, 5, 10, and 15. 10 items were scored out of 100, with higher scores indicating higher ability to perform activities of daily living.
4. The levels of serum bone metabolic markers and inflammatory mediators were compared before and after treatment in the three groups: patients were instructed not to eat or drink after 22 : 00 on the first day before the test, and 5 ml of venous blood was drawn in the early morning of the second day on an empty stomach for the test. We measured the levels of bone metabolism markers such as cartilage oligomeric matrix protein (COMP), type II collagen carboxy-terminal peptide (CTX-II), matrix metalloproteinase-3 (MMP-3), and serum inflammatory mediators such as interleukin-1*β* (IL-1*β*), tumor necrosis factor-*α* (TNF-*α*), and hypersensitive C-reactive protein (hs-CRP) by enzyme-linked immunosorbent assay (ELISA), Serum COMP ELISA Kit, Serum CTX-II ELISA Kit, Serum MMP-3 ELISA Kit, Serum IL-1*β* ELISA Kit, Serum TNF-*α* ELISA Kit, and Serum hs-CRP ELISA Kit which were purchased from Shanghai Xitang Biotechnology Co. The specific operation steps were carried out in accordance with the instructions of the ELISA kit.

### 2.7. Judgment of Efficacy

The efficacy criteria were developed with reference to the “Guidelines for Clinical Research of New Chinese Medicine (Trial)” [10] and combined with knee X-ray examination. ① After treatment, the patient's clinical symptoms and signs mostly disappeared, the joint movement returned to normal, the X-ray indicated that the joint returned to normal, and the LKS score increased by more than 90% and was considered as healed. ② The patient's symptoms and signs improved significantly, and he/she could carry out normal life and work, the X-ray film indicated that the joint pathology was significantly improved, and the LKS increased by 71% to 90% and was considered as marked effect. ③ The patient's symptoms and signs were relieved after treatment, but the joint movement was still limited to a certain extent, the X-ray showed some improvement of the joint pathology, and an increase of 31% to 70% in the LKS was considered as valid. ④ The patient's clinical symptoms and signs did not improve after treatment, his/her daily life was limited, X-rays showed no improvement in the joint pathology, and the LKS increased by less than 31% and was considered as invalid. Excellent rate = number of (healed + marked effect) cases/total number of cases × 100%.

### 2.8. Statistical Method

All data were processed with SPSS 22.0 statistical software, and GraghPad prism 8 was used to make statistical graphs. The count data was expressed as case, %, and chi-square (*χ*^2^) test was performed. The measurement data were tested according to normality, *t*-test was used between two groups conforming to normality, and One-Way ANOVA (*F*-test) was used between multiple groups, expressed as mean ± standard deviation (mean, (SD)). *P* < 0.05 indicated that the difference was statistically significant.

## 3. Results

### 3.1. Comparison of Clinical Efficacy

After 4 weeks, 14 cases (35.00%) were healed, 15 cases (37.50%) were marked effect, 9 cases (22.50%) were valid, and 2 cases (5.00%) were invalid in treatment group 1, with an excellent treatment rate of 72.50%. There were 10 cases (25.00%) healed, 10 cases (25.00%) with marked effect, 15 cases (37.50%) with valid effect, and 5 cases (12.50%) with invalid effect in treatment groups 2, with an excellent treatment rate of 50.00%. In the joint group, 23 cases (57.50%) were healed, 13 cases (32.50%) were marked effect, 4 cases (10.00%) were valid, and 0 cases were invalid, with an excellent treatment rate of 90.00%. We conducted a statistical analysis of the excellent rates of treatment in the three groups. The results showed that the excellent efficacy rate of the three groups was as follows: joint group > treatment group 1 > treatment group 2, and the difference between any two groups was statistically significant (*P* < 0.05) (Figure 1).

### 3.2. Comparison of VAS, LKS, and ADL Scores before and after Treatment

There was no significant difference in the scores of VAS, LKS, and ADL in the three groups before treatment (*P* > 0.05). The VAS scores decreased and Lysholm scores and ADL scores increased in all three groups after treatment (*P* < 0.05). Among them, the VAS scores were as follows: joint group < treatment group 1 < treatment group 2, and the difference between any two comparisons was statistically significant (*P* < 0.05). The Lysholm scores and ADL scores were as follows: combined group < treatment 1 group < treatment 2 group, and the difference between any two comparisons was statistically significant (*P* < 0.05) (Figure 2).

### 3.3. Comparison of Serum Bone Metabolism Marker Levels before and after Treatment

The differences in the levels of serum COMP, CTX-II, and MMP-3 in the three groups before treatment were not statistically significant (*P* > 0.05). In contrast, the levels of serum COMP, CTX-II, and MMP-3 decreased significantly in all three groups after treatment (*P* < 0.05). The levels of the above indexes in the joint group were lower than those in treatment groups 1 and 2, while treatment group 1 was lower than treatment group 2, and the difference was statistically significant (*P* < 0.05) (Figure 3).

### 3.4. Comparison of Serum Inflammatory Mediator Levels before and after Treatment

There was no statistically significant difference in the pretreatment levels of serum IL-1*β*, TNF-*α*, and hs-CRP among the three groups (*P* > 0.05). After treatment, serum IL-1*β*, TNF-*α*, and hs-CRP levels decreased in all three groups (*P* < 0.05). Among them, the levels of serum IL-1*β*, TNF-*α*, and hs-CRP in the joint group were lower than those in treatment group 1 and treatment group 2, while the levels of the above indexes in treatment group 1 were lower than those in treatment group 2, and the differences were statistically significant (*P* < 0.05) (Figure 4).

### 3.5. Safety

The three cohorts underwent routine blood, urine, and stool tests, liver and kidney function tests, and electrocardiograms before and after treatment, and none of the results were significantly abnormal. No severe skin itching, red rash, or burns were observed in any of the patients treated with Tongluozhitong prescription dip-soaking therapy, which indicates that Chinese medicine treatment, western medicine treatment, and combined treatment regimens have a good safety profile.

## 4. Discussion

Total knee arthroplasty is the best treatment for patients with end-stage KOA, but this surgical treatment can be traumatic to the patient's body and has the disadvantages of high cost and high risk of postoperative infection. Therefore, effective options to delay or even reverse the degenerative changes in the knee joint before the patient's disease becomes advanced are always the key to clinical treatment [11, 12]. The pathogenesis of the disease is not fully understood, and numerous studies [13, 14] have shown that inflammatory factors play an important role in the production of KOA. IL-1*β* and TNF-*α* are common inflammatory cytokines with multiple biological functions, both of which can induce the synthesis of matrix metalloproteinases (MMPs), thereby increasing the degradation of chondrocytes and eventually leading to the destruction of articular cartilage and the formation of osteoarthritis. In addition, TNF-*α* can also damage cartilage and stimulate chondrocytes by stimulating the production of prostaglandin E2 by anterior synovial cells, causing them to release large amounts of fibrinolytic activators and ultimately aggravate joint damage by converting fibrinogen [15].

The KOA patients included in the study were treated with dip-soaking of Tongluozhitong prescription, sodium hyaluronate injection, and a combination of both, respectively. The results showed that the clinical efficacy of treatmen group 1 was significantly higher than that of treatment group 2, and the improvement of pain, joint function, and activity scores and serum inflammatory factors were significantly better in treatment group 1 than in treatment group 2 after treatment, while, compared with these two groups, the joint group showed better efficacy and improvement in each index. Currently, sodium hyaluronate is a commonly used drug in the clinical treatment of KOA patients. The decreased synthesis of hyaluronic acid by the synovial membrane in patients with KOA can lead to damage to knee cartilage. Thus, intra-articular injection of exogenous sodium hyaluronate into the knee joint cavity can increase the content of macromolecular hyaluronic acid to restore the viscoelasticity of the joint fluid and reconstruct the articular cartilage. In addition, this drug can inhibit the release of inflammatory mediators to eliminate swelling symptoms, reduce joint pressure and cartilage friction, and delay arthrosis [16]. Chinese medicine dip-soaking therapy has also been gradually applied to the treatment of KOA in recent years, and its mechanism of action in the treatment of KOA is divided into two main aspects [17, 18]. The first is the efficacy of the drugs themselves; the drugs used in herbal dip-soaking can be selected according to the patient's disease evidence and specific performance. Among the drugs selected in this study, myrrh and frankincense have the function of invigorating blood, promoting qi, dredging collaterals, and relieving pain; garden balsam stem has the effects of dispelling wind and dampness, relaxing muscles and activating blood, and detoxifying and relieving pain; *Zanthoxylum bungeanum* Maxim. warms the middle and disperses cold to relieve pain, and radix puerariae is cold-natured, which can avoid excessive pungency and warmth in the whole prescription. The whole prescription has the effects of dispelling wind and dampness, promoting blood circulation and dredging collaterals, dispelling cold, and relieving pain. The second is the warming effect produced by the heating of the drug. The efficacy of the drug combined with the heat can promote the expansion of blood vessels in the affected area and accelerate blood circulation, so that the drug can reach the lesion directly through the expanded pores and thus play a therapeutic role. Modern pharmacological studies have confirmed that myrrh [19], frankincense [20], and *Zanthoxylum bungeanum* Maxim. [21] have strong anti-inflammatory effects, in addition to significant analgesic effects; the dip-soaking therapy of Tongluozhitong prescription takes into account anti-inflammatory and pain-relieving effects and treats the root of the disease, which is more conducive to the relief of patients' symptoms. Tongluozhitong prescription treats the root cause by exerting the effect of dispersing cold and relieving pain, activating blood circulation, and treating the symptoms by nourishing and moisturizing anti-inflammation with sodium hyaluronate. The combination of the two drugs achieves the purpose of treating both principal and secondary aspects of disease so that the combination of herbal collapse treatment can lead to further improvement in the clinical outcome of KOA patients. However, as most KOA patients are middle-aged and elderly, they are susceptible subjects and should be closely monitored during treatment, with continuous improvement of the formula, enhanced communication between doctors and patients, and timely management of adverse reactions during treatment to improve treatment effectiveness.

COMP, CTX-II, and MMP-3 are all markers of cartilage metabolism. COMP is a component of cartilage noncollagenous protein and is a sensitive indicator for clinical evaluation of the degree of articular cartilage damage, and an increase in its level usually indicates increased damage to knee cartilage [22]. CTX-II is a small molecule peptide produced by the stimulation of type II collagen by protease, and its level reflects the degradation ability of type II collagen, which is involved in the degeneration of articular cartilage and the formation of osteoarthritis [23]. MMP-3 is mainly secreted by chondrocytes and synovial cells, and its expression level is closely related to articular cartilage damage and can be used as a sensitive indicator for the diagnosis of osteoarthritic conditions [24]. In this study, the levels of COMP, CTX-II, and MMP-3 were significantly lower in the joint group after treatment than in the other two groups, while treatment 1 group was lower than treatment 2 group. It is suggested that the dip-soaking therapy of Chinese medicine is more effective in regulating the bone metabolic index of KOA patients to slow down the process of articular cartilage degeneration, and the combination of Chinese medicine dip-soaking therapy is an effective solution in the clinical treatment of patients with KOA, or patients with low tolerance to multiple solutions can be treated with herbal impregnation, which can also achieve better therapeutic results.

## 5. Conclusion

In a word, the dip-soaking therapy of Tongluozhitong prescription is more advantageous than intra-articular sodium hyaluronate injection treatment in suppressing the level of serum bone metabolic markers and inflammatory mediators, reducing pathological joint damage, relieving symptoms of pain, alleviating degenerative joint symptoms, and improving knee function in KOA patients. The combination of the two in KOA patients can significantly improve the efficacy and has a good safety profile.

## Figures and Tables

**Figure 1:** Comparison of clinical efficacy between treatment group 1, treatment group 2, and joint group. Excellent rate: compared with treatment group 1,  ^∧^*P* < 0.05; compared with treatment group 2, ^*∗*^*P* < 0.05.

**Figure 2:** Comparison of VAS, LKS, and ADL scores before and after treatment between treatment group 1, treatment group 2, and joint group. (a) Mean VAS scores. (b) Mean LKS scores. (c) Mean ADL scores. Compared to the same group before treatment, ^#^*P* < 0.05; compared with treatment group 1 in the same time period, ^∧^*P* < 0.05; compared with treatment group 2 in the same time period, ^*∗*^*P* < 0.05.

**Figure 3:** Comparison of serum bone metabolism marker levels before and after treatment between treatment group 1, treatment group 2, and joint group. (a) Mean COMN levels. (b) Mean CTX-II levels. (c) Mean MMP-3 levels. Compared to the same group before treatment, ^#^*P* < 0.05; compared with treatment group 1 in the same time period,  ^∧^*P* < 0.05; compared with treatment group 2 in the same time period, ^*∗*^*P* < 0.05.

**Figure 4:** Comparison of serum inflammatory mediator levels before and after treatment between treatment group 1, treatment group 2, and joint group. (a) Mean IL-1*β* levels. (b) Mean TNF-*α* levels. (c) Mean hs-CRP levels. Compared to the same group before treatment, ^#^*P* < 0.05; compared with treatment group 1 in the same time period, ^∧^*P* < 0.05; compared with treatment group 2 in the same time period, ^*∗*^*P* < 0.05.

**Table 1:** Comparison of basic information of treatment group 1, treatment group 2, and joint group.

Information		Treatment group 1 (*n* = 40)	Treatment group 2 (*n* = 40)	Joint group (*n* = 40)	*P* value
Gender (case, %)	Male	17 (42.50)	18 (45.00)	16 (40.00)	0.903
	Female	23 (57.50)	22 (55.00)	24 (60.00)	

Lesion site (case, %)	Unilateral	26 (65.00)	28 (70.00)	29 (72.50)	0.761
	Bilateral	14 (35.00)	12 (30.00)	11 (27.50)	

Age, mean (SD), years		53.96 ± 7.26	54.35 ± 8.01	54.12 ± 7.46	0.974
Disease duration, mean (SD), years		3.29 ± 1.29	3.18 ± 1.38	3.24 ± 1.34	0.934

## Data Availability

The datasets used and/or analyzed during this study are available from the corresponding author upon reasonable request.
